# Resilient Public Transport Construction in Mega Cities from the Perspective of Ecological Environment Governance

**DOI:** 10.1155/2022/9143618

**Published:** 2022-08-08

**Authors:** Wenjing Ge, Guixiang Zhang

**Affiliations:** School of Urban Economics and Public Administration, Capital University of Economics and Business, Beijing 100070, China

## Abstract

With the rapid development of the social economy, environmental and resource constraints of economic growth are becoming more and more serious. Therefore, for cities, we should take the road of green development and sustainable development. On the one hand, we should fully implement the basic policies issued by the central government. On the other hand, we should fully integrate the actual situation of the city to make it better implemented, which will help to improve the ability of ecological environment governance and consolidate the ecological advantages of the city. With the development of the urban economy and the continuous increase of population, the development pressure faced by cities is also increasing. Innovating urban construction mode has increasingly become the focus of the development of the new era. The main reason is that the continuous growth of the urban population, environmental pollution, traffic congestion, and ecological damage has caused great trouble to urban residents. The traditional public service governance model has been unable to meet the current public service needs of urban residents. Based on this background, major cities around the world have begun to study urban resilience in order to prevent and resist the interference and impact brought by the outside world and maintain the sound development of the urban system. Based on the demand for ecological environment governance, this study analyzes the current situation and causes of urban ecological environment governance in China and the problems existing in urban resilient transportation construction in China, and puts forward corresponding countermeasures for ecological environment governance and the current situation of urban resilient public transportation construction. This study has great theoretical and practical significance to promote the sustainable development of the Chinese ecological environment and the resilience construction of urban transportation.

## 1. Introduction

Lu Xinyuan, vice president of the China Environmental Science Association, said in his 2012 visit report that since 1996, the incidence of environmental mass events in China has increased at an average annual rate of 29%, and environmental problems have become the fastest-growing disease of concern to our people [1]. Recently, Chai Jing, a famous female reporter for CCTV who has left her job, made a documentary entitled “under the dome” at her own expense, which aroused people's extensive attention and discussion on urban ecological and environmental problems and the harm to the environment to the human body [2]. Environmental problems have become major living, economic and political problems that our country and people must face and deal with [3]. At present, the environmental problems in Chinese cities mainly include exhaust pollution, acid rain, photochemical smoke, greenhouse effect, dust sandstorm, building noise, car noise, and electromagnetic field pulse radiation. Even more serious concerns are plastic bag pollution, battery pollution, and wastewater discharge.

In the report of the Third Plenary Session of the 18^th^ CPC Central Committee, “ecological civilization” appeared three times in total, and the conference clearly proposed to delimit the “ecological red line,” which reflects the great importance attached by the party and the state to ecological civilization [4]. In recent years, a series of urban problems such as smog, drinking water pollution, noise pollution, population explosion, and greenhouse effect caused by excessive carbon emissions have been highlighted in the public's vision. In order to alleviate and solve the urban ecological environment problems in the process of urbanization, it is imperative to explore and study the urban ecological environment governance [5]. As can be seen from the chart, China's cities with high carbon emissions are big cities like Jinan, Shanghai, and Guangzhou, mainly because there are too many means of transportation in big cities, while China's second-and third-tier cities have relatively small carbon emissions.

Figure 1 shows the total carbon dioxide emissions of 30 cities in China from 2007 to 2016. Public transport has the greatest impact on the urban ecological environment because urban development is accompanied by disaster risks [6]. In recent years, more and more attention has been paid to the sustainable development of the transportation industry and environmental protection [7]. The current complex and diverse transportation problems show that the original comprehensive transportation system can not meet the transportation power strategy and the goal of green development. Therefore, people are more inclined to find ways to build sustainable transportation. Ecological transportation has gradually come into people's sight, which has aroused heated discussion among scholars from all walks of life [8]. As can be seen from the figure, China's megacities, such as Shenzhen, Shanghai, and Beijing, have good green transportation construction, but compared with 2018, they show a downward trend. With the decline of urban scale, the construction intensity of urban green transportation has also shown a decreasing trend, which is directly related to the economic development intensity of the city.

Figure 2shows the construction of green transportation in various types of cities in China. The development of any work in China needs the support of the system, and the implementation of the system needs the cooperation of corresponding departments [9]. The governance of the urban ecological environment is a “thorny” problem involving the comprehensive governance of multiple departments [10]. Moreover, in the process of urban ecological environment governance in China, due to various factors inside or outside the system, The governance of the urban ecological environment basically presents a state of “fragmentation,” and the tenacity governance theory is to solve the problems of “fragmentation” and “thorny.” This kind of “thorny” and “fragmentation” in China's urban ecological environment governance just coincides with the theory of holistic governance [11]. Therefore, based on the needs of ecological environment governance, this study analyzes the current situation and causes of urban ecological environment governance and the problems existing in urban resilient transportation construction in China and puts forward corresponding countermeasures for the current situation of ecological environment governance and urban resilient public transportation construction. It is of theoretical and practical significance to explore the theory of resilience governance to solve the strategy of urban ecological environment governance road and urban public transportation construction in China.

## 2. Theoretical Research

### 2.1. Overview of the Connotation of Urban Toughness

From the perspective of origin, the word toughness originated from Latin (resilio), which means the ability to reset an object to its original state. With the development of society, the concept of resilience has been applied to various fields [12]. In engineering, with the development of western industrial technology, scholars use toughness to express the recovery ability of an object after deformation or injury under the action of the outside world; In psychology, resilience is used to describe resilience after mental or psychological setbacks. By the end of the 20th century, with the popularity of the concept of resilience in the research and development of various disciplines, the concept of resilience has been gradually applied to many disciplines, such as ecology, economics, sociology, geography, psychology, and engineering. The understanding, research, and application of resilience in various disciplines are also very different as shown in Table 1 [13].

Resilience has the characteristics of dynamic and collaborative evolution. As a necessary element of urban high-quality development, its concept has been widely used in urban development and evolved into “urban resilience” [14]. Urban resilience refers to the ability of a city to operate normally and smoothly under the interference of uncertain factors in its development and quickly recover to its initial state when impacted. In the development of urban resilience, different scholars in different countries have conducted different scientific research on urban resilience. Through analysis and research, the resilience alliance points out that the development of urban resilience mainly includes four aspects: urban social resilience, urban engineering resilience, urban ecological resilience, and urban economic resilience. Urban Engineering resilience describes that the perfect urban infrastructure construction provides a solid guarantee for the development of urban resilience. It can effectively prevent or reduce disasters when disasters come [15]. At the same time, accumulating experience can optimize urban engineering resilience to reduce the risk brought by such disasters [16]. Urban ecological resilience describes the ability of the urban ecosystem to recover to its original state when subjected to sudden and uncertain interference or impact, mainly including the resistance of the urban ecosystem to natural disasters, adaptation to natural changes in ecosystem, and so on. Urban economic resilience describes the ability of the urban economy to return to its original state when it is subjected to external interference and impact. To sum up, urban resilience is the ability of a city to operate its urban system normally in the face of uncertain and unknown interference or impact [17].

### 2.2. Theoretical Research on Ecological Environment Governance

“Governance” comes from Latin and ancient Greek. It originally means control, guidance, and manipulation. It has been applied to economics, politics, sociology, and other fields. It is generally believed that Rosenau is the main founder of governance theory. His representative works are governance in the 21^st^ century and governance without government [18]. He believes that governance is a regulatory mechanism, which can play an effective role even without formal authorization. “Unlike governance, governance refers to an activity supported by common goals. The main body of these management activities may not be the government, nor does it need to rely on the coercive force of the state.” As an authoritative scholar of governance theory, Gerry stoke believes that governance is a new development direction of government rule [19]. It includes not only government mechanisms, but also non-governmental mechanisms. Ecological environment control includes air pollution prevention and control, soil environment comprehensive control, forest area ecological restoration and wetland protection, desertification prevention and control, soil erosion prevention and control, and so on. Ecological environment governance is a strategic decision put forward by China to protect and build the ecological environment and realize sustainable development. Mainly through carrying out trees and grass, soil erosion control, desertification control, ecological agriculture, and other ways, the construction of beautiful mountains and rivers of the motherland.

In the theory of ecological environment governance, structural functionalism is an important branch. Parsons, an American sociologist, is the leader of the school of structural functionalism. His structural-functional analysis focuses on the mechanism of promoting the stability and order of the social system. He believes that a complete system should have four functions: adaptation, goal realization, integration, and mode maintenance, as shown in Figure 3.

In ecological environment governance, simple cross-border cooperation cannot constitute holistic governance. To distinguish whether a government's management form is holistic, the government needs to judge from the degree of relationship between the two dimensions of objectives and means [20]. According to whether the policy objectives and means of the organization are mutually beneficial, the governance forms of the government are divided into five types: progressive government, Lord government, overall government, fragmented government, and collaborative government, as shown in Figure 4.

From the perspective of urban ecological environment governance, we can analyze the above five forms of government governance in this way. In progressive government governance, driven by the interests of regions and departments, before the evaluation of superior departments, all departments and regions do not communicate with each other and act in their own way. It can be said that their objectives are conflicting in their respective areas of jurisdiction. However, when facing some joint problems, they have to cooperate. In this case, due to the limitations of regional scale and departmental interests, it is difficult to form a centralized overall governance strategy for urban ecological environment governance.

## 3. Ecological Environment Problems Existing in Mega Cities in China and the Current Situation of Resilient Transportation Construction

### 3.1. Problems and Causes of Urban Ecological Environment Governance in China

#### 3.1.1. Control Fragmentation

The fragmentation of governance function means that under the joint topic of urban ecological environment governance, the relevant functional departments have not achieved the overall governance effect of mutual coordination. In China, as the main body of urban ecological environment governance, the government should use policy, system, economy, culture, law, and other means to achieve mutually reinforcing effects on the goal orientation and means of urban ecological environment governance. However, in reality, due to the division of functional departments, the goals and means can not echo each other. On the whole, China is not only a developing country but also the country with the largest population in the world. The per capita economic strength is still a certain distance from that of western developed countries. Especially in the past few decades, the primary task of governments at all regions and levels is almost to develop the economy, and the economic development of many places is almost at the cost of destroying the balance of the urban ecological environment.

#### 3.1.2. Insufficient Participation of the Public and Other Governance Subjects

The subjects of urban ecological environment governance include government, citizens, enterprises, and environmental NGOs. Although the government plays a leading role in this system, the role of other governance subjects can not be ignored. However, due to the influence of various internal and external factors, the participation and role of citizens, enterprises, environmental NGOs, and other non-governmental governance subjects in China's urban ecological environment governance are not high and obvious. The environmental NGO project was established by China Development Bulletin for environmental NGOs, which is supported by the Ford Foundation and has an advisory committee composed of representatives from China Environmental NGOs as the consultants of the project. By the end of February 2015, the State Administration for Industry and Commerce of the people's Republic of China announced that the number of enterprises in China was 18.7149 million, while the data of the Ministry of environmental protection showed that from 2007 to 2014, only 14665 enterprises in China had obtained environmental mark certification, including some enterprises with invalid environmental mark certification, which is the tip of the iceberg compared with the number of enterprises actually registered in China, It is far from western developed countries.

#### 3.1.3. The Management Mode Is Rigid and Outdated

At this stage, China implements a management system in which governments at all levels are responsible for local environmental quality, environmental protection administrative departments implement unified supervision and management, and relevant departments implement supervision and management, that is, the management mode of direct control by the government. Under this model, the governance of the urban ecological environment means that the government should directly invest a lot of financial and material resources. The governance of the urban ecological environment is a long-term and expensive project, and the long-term financial expenditure of the government is inevitably unable to support it. The mode of direct government control means the excessive use of administrative means. Although administrative means have the characteristics of being fast, efficient, compulsory and authoritative, their effects are not long-term. The excessive use of administrative means by the government is not only not conducive to the good absorption and utilization of social resources in urban ecological environment governance, but also consumes too many administrative resources, reducing the social recognition of environmental management. This is in contradiction with the persistence of urban ecological environment governance.

#### 3.1.4. Causes of Urban Ecological Environment Governance Problems in China

The self-interest characteristics of the government. The school of public choice theory represented by Buchanan brings the behavior of the government and government staff into the hypothesis of “economic man,” and believes that the government and government staff have a self-interest orientation. They pursue the maximization of individual interests. When the public interests conflict with their own interests, they choose their own interests more. At present, the important measurement standard for the assessment and selection of officials in China is GDP. Even if there are assessment indicators such as people's livelihood improvement, social progress, and ecological benefits, GDP still occupies the main position, which is easy to lead the local government and officials to reduce the standard of environmental access and introduce some enterprises with high pollution and high energy consumption at the cost of destroying the environment and natural resources in order to promote the economic growth of their jurisdiction, Turn a blind eye to their pollution and destruction, and even interfere with the law enforcement of the environmental department.

### 3.2. Problems in Urban Traffic Toughness Construction

Generally speaking, the basic meaning of resilience is to effectively mitigate the impact of external shocks, maintain the operation of main functions, and quickly recover from the crisis. At present, the problems existing in the construction of urban resilient transportation include the following aspects.

#### 3.2.1. Serious Traffic Pollution

The increasing development of the social economy has brought about the rise in car ownership and the increase in exhaust emissions. The resulting environmental and noise pollution has become an important problem faced by many cities, which will not only interfere with people's normal life and work but also affect everyone's health. Automobile exhaust contains carbon dioxide, sulfur dioxide, and nitrogen oxides, which aggravates the deterioration of the greenhouse effect and destroys the ecological environment.  Table 2 shows the carbon emission factors of main automobile fuels. According to the table, among all fuels, natural gas has the highest carbon emission factor, at 99%, followed by kerosene and fuel oil, while gasoline and diesel are also relatively high, at 98% and 98.2%, respectively. Traffic noise pollution is an important part of urban noise pollution. The noise brought by the subway and expressway makes many surrounding residential areas seriously affected by traffic noise. According to statistics, environmental noise exposure from road traffic and other sources seriously endangers health. It is estimated that at least 1 million healthy life years are lost in Western Europe every year, mainly due to sleep disorders, troubles, and cardiovascular diseases.

#### 3.2.2. Road Traffic Congestion

The transportation network undertakes the function of urban transportation distribution, promotes regional economic development, and greatly improves the efficiency of urban operation. In recent years, Fujian Province has strengthened road reconstruction and vigorously built expressways, which has alleviated the traffic pressure to a certain extent. However, the traffic congestion problem caused by holidays and morning and evening peaks is still significant. The daily congestion period is mainly concentrated in the morning and evening peaks, which will last for 2 hours or even longer. The main reason is that the central urban area undertakes a large number of residents and jobs in a small area, and the business district is mostly concentrated in important sections of the central area. The parking lot is in short supply and the “one in one out” parking mode aggravates the traffic congestion. In addition, the illegal parking of motor vehicles and the occupation of motor vehicle lanes by electric vehicles increase the probability of accidents, which is also one of the reasons for traffic congestion.  Figure 5 shows the variation coefficient of ecological traffic efficiency of China's megacities from 2007 to 2016. Traffic congestion not only affects people's normal travel but also causes great resistance to social development and the environment. Delays, excessive fuel consumption, and higher vehicle emissions caused by traffic congestion are the deep-seated effects of traffic congestion, which have caused huge economic losses to the transportation system.

## 4. Countermeasures for Improving Urban Ecological Environment Governance Capacity and Urban Resilient Traffic Construction

### 4.1. The Urban Development Planning Is Scientific and Reasonable

For cities, coordinated development is very important. If there is a large gap in the economic level of regional development of a city, there will be great differences in its ecological construction; At the same time, there will be some differences between urban ecological construction and township ecological construction. The existence of these differences will mean that urban green construction cannot be carried out uniformly, and it is difficult to form an urban ecological circular economy. Based on this, urban development planning should reflect scientificity and rationality, adjust the ecological plan against the background of economy and society, focus on solving the problem of inconsistency in urban planning, and carry out ecological construction in different areas; At the same time, fully combine the central top-level design and the specific practice of the city, and integrate the ecological environment governance into all aspects of social construction based on the SWOT analysis framework. The SWOT analysis framework is shown in Figure 6. SWOT analysis is a method to systematically evaluate the various factors, so as to select the best business strategy. Therefore, SWOT analysis is actually a way to synthesize and summarize all aspects of the internal and external conditions of an enterprise, analyze its advantages and disadvantages, opportunities and threats, and then help enterprises to make strategic choices.

### 4.2. Improve Laws and Regulations on Urban Ecological Environment Governance

In order to pursue economic interests, some industrial enterprises have not attached great importance to the specific requirements of ecological construction. Although the cities have taken regulatory measures and investigated them one by one, it is difficult to avoid omissions. Based on this, the legal and regulatory system of urban ecological environment governance should be further improved. Taking Shaanxi Province as an example, by 2019, the province had issued 23 environmental protection standards, including the emission control standard of volatile organic compounds, the comprehensive sewage discharge standard of the Yellow River Basin in Shaanxi Province, the emission standard of air pollutants for key industries in Guanzhong area, the emission standard of air pollutants for boilers, and the emission standard of water pollutants for rural living sewage treatment facilities, including nine pollutant emission (control) standards.

### 4.3. Pay Attention to the Development of Green Travel Mode

Ecological transportation emphasizes the low-carbon, ecological, and green environmental protection of travel mode, which needs to meet the harmonious development of nature, economy, and society. Therefore, urban traffic construction must focus on green development, uphold the concept of sustainability, and reduce the negative impact on the environment, such as exhaust emission and noise pollution, on the basis of meeting people's travel needs. At the same time, when carrying out transportation planning and construction, we must realize that land resources are limited, reasonably plan urban land and adjust measures to local conditions. Eco city transportation needs to actively develop and use new energy vehicles, such as trams, taxis, and electric buses, encourage and guide people to use new energy vehicles, and improve charging piles and other facilities. Using new energy vehicles as the main body instead of motorized travel mode is conducive to reducing air pollution, saving resources, and promoting the development of sustainable transportation.  Table 3 shows the potential for energy conservation and emission reduction in cities.

### 4.4. Building a Green and Resilient Transportation System

To build a transportation system with public transport as the main body and establish a perfect public transport system, we should strive to form a functional level perfect urban public transport structure system with public transport as the framework, conventional public transport as the basis, and various modes as the supplement, and improve the public transport service facility system. On the other hand, public transport stations should do a good job in the slow connection channel, solve the transfer problem to the greatest extent, improve the service level and attractiveness of public transport, and reduce the travel distance of residents. Finally, it is necessary to appropriately increase or reduce the departure frequency and the number of buses according to the traffic travel needs of different periods and regions and set the phase of bus lanes and special signals to ensure bus priority and improve the efficiency of public transport.

## 5. Conclusion

The construction and rapid development of resilient urban transportation promote the rapid development of urbanization, which not only facilitates people's travel but also better promotes communication between cities as a link connecting various urban districts. However, with the rapid development of urbanization, there is a contradiction between people's demand for high-quality life and the limitation of urban resources. The traditional demand-oriented development model has been unable to meet the severe traffic problems. The disorderly development within the city makes the coordinated development of the region difficult and slow, which runs counter to the requirements of green development and the construction of a beautiful China. Based on the demand for ecological environment governance, this study analyzes the current situation and reasons for urban ecological environment governance in China and the problems existing in the construction of urban resilient transportation in China. Based on this, this study puts forward the countermeasures to optimize the urban ecological environment governance mode and build the urban resilient transportation system. This study has important reference significance for promoting the sustainable development of green transportation and urban transportation.

## Figures and Tables

**Figure 1:** Total carbon dioxide emissions of 30 cities in China from 2007 to 2016.

**Figure 2:** Construction of green transportation in various types of cities in China.

**Figure 3:** Parsons' functional analysis model.

**Figure 4:** Relationship between objectives and means.

**Figure 5:** Average and coefficient of variation of national urban traffic efficiency.

**Figure 6:** SWOT analysis framework diagram.

**Table 1:** Evaluation index of urban toughness.

Target level and index level	Secondary index layer	Unit and nature	Index meaning
Urban infrastructure resilience	Urban road area per capita (XS)	M2/person (+)	Traffic accessibility
	Urban construction land area (XG)	Square kilometers (+)	Land use
	Length of drainage pipe (XM)	Km (+)	Infrastructure construction
	Per capita domestic water consumption x1)	Ton/person (−)	Water resources supply
	Per capita power consumption (xn)	KWh/person (−)	Power supply
	Total LPG supply (x13)	Ton (−)	LPG supply
	Number of internet broadband access users (x14)	Household (+)	Network popularity

Urban ecological resilience	Per capita green area (xis)	M2/person (+)	Urban environmental level
	--Comprehensive utilization rate of general industrial solid waste (x16)	% (+)	Comprehensive utilization level of waste
	Centralized treatment rate of sewage treatment plant (x1)	% (+)	Sewage treatment intensity
	Greening coverage rate of built-up area x1)	% (+)	Urban greening level
	Harmless treatment rate of domestic waste (x19)	% (+)	Environmental pollution control ability

Urban economic resilience	Public revenue (xn)		10000 yuan (+)
	Financial revenue status		

Amount of foreign capital actually used in the current year (X21)	USD 10000 (+)	Dependence on foreign capital utilization	
	Resident RMB savings deposit balance (x2)	10000 yuan (+)	Resident financial capital
	GDP per capita (x2)	Yuan/person (+)	Total economic development
	Proportion of secondary industry in GDP (x24)	% (+)	Economic structure
	Proportion of tertiary industry in GDP (X2S)	% (+)	Economic structure
	Public expenditure (XX)	10000 yuan (−)	Financial input
	RMB deposit balance of financial institutions at the end of the year (xn)	10000 yuan (+)	Capital reserve capacity
	Balance of RMB loans of financial institutions at the end of the year (XX)	10000 yuan (−)	Capital lending capacity
	Total retail sales of social consumer goods (X29)	10000 yuan (+)	Consumption capacity
	Per capita investment in fixed assets (cx3o)	Yuan/person (+)	Investment level

**Table 2:** Carbon emission factors of main fuels.

Fuel	Carbon	Gasoline	Kerosene	Diesel oil	Fuel oil	Natural gas
CCF	27.28	18.9	19.6	20.17	21.09	15.32
HE	192.14	448	447.5	433.3	401.9	0.384
COF (%)	92.3	98.0	98.6	98.2	98.5	99.0

**Table 3:** Energy conservation and emission reduction potential in all cities of China.

City	Energy saving potential	Emission reduction potential
Beijing	0.26	0.65
Tianjin	0.14	0.22
Shijiazhuang	0.21	0.27
Taiyuan	0.11	0.18
Hohhot	0.15	0.2
Shenyang	0.19	0.4
Changchun	0.12	0.28
Harbin	0.09	0.15
Shanghai	0.35	0.52
Nanjing	0.12	0.39
Hangzhou	0.03	0.28
Hefei	0.01	0.27
Fuzhou	0.08	0.11
Nanchang	0.11	0.25
Jinan	0.13	0.52
Zhengzhou	0.25	0.34
Wuhan	0.04	0.21
Changsha	0.03	0.19
Guangzhou	0.19	0.53
Nanning	0.08	0.18
Haikou	0.02	0.17
Chongqing	0.05	0.13

## Data Availability

The labeled dataset used to support the findings of this study are available from the corresponding author upon request.
